The article "Case series on testicular torsion: an educational emergency for sub-Saharan Africa" was published in 2013. Journal: Pan Afr Med J.

# Case series on testicular torsion: an educational emergency for sub-Saharan Africa

**DOI:** 10.11604/pamj.2013.14.18.1736

**Published:** 2013-01-12

**Authors:** Evarist Baruga, Ian Guyton Munabi

**Affiliations:** 1 Senior Consultant Surgeon of Private Hospitals in Kampala, Director of Wandegeya Medical center. P.O. Box 11257 Kampala, Uganda; 2 Department of Human Anatomy, School of Biomedical Sciences, Makerere University College of Health Sciences. P.O. Box 7072 Kampala, Uganda

**Keywords:** Human, male, spermatic cord torsion, surgery, diagnosis, education, etiology, differential diagnosis

## Abstract

Testicular torsion remains a common surgical emergency of adolescent males presenting with sudden onset of intense scrotal pain in Africa. While the magnitude of testicular torsion is not known it has been identified as a cause of male infertility. Testicular loss in Africa is directly related to delay in surgery and the referral patterns at the point of first contact with health workers. This paper sets out to demonstrate the importance of the patient's age in the diagnosis of testicular torsion. A surgical audit was made of patients records collected over the last 30 years, for presentation of testicular related symptoms and analyzed to identify changes in the patterns of diagnosis over time and in different countries. There were 305 records found, for patients with an age range of 9-56 years. There were 195/305 (64%) with orchitis and 110/305 (36%) with testicular torsion. Testicular torsion is more common under the age of 18 years while orchitis was more common after 18 years of age (rho = -0.834, p value > 0.001 one tailed). This paper supports the development of educational interventions that promote the use of age in a simple diagnostic rule of the thumb for communities and lower cadre health workers in low resource settings.

## Introduction

Testicular torsion is a common surgical emergency of adolescent males presenting with sudden onset of intense scrotal pain [1]. Anatomically testicular torsion follows a congenital anomaly in predisposed individuals that allows the testis to rotate, twisting the spermatic cord, resulting in loss of blood supply and eventual testicular necrosis [2]. Patients usually present with acute onset of severe scrotal pain, with or without a history of trauma in males under the age of 18 years. The extent of testicular rotation determines the time to total testicular loss. Since the anomaly is commonly bilateral definitive management requires early identification by the first contacted health worker followed by prompt surgical intervention.

According to Kapoor, one in every 4000 males under the age of 25 years develops testicular torsion annually. This happens mostly in the colder months of the year. [1] On the African continent the magnitude of testicular torsion is not known though according to Ekwere et al, testicular torsion was the cause of male infertility in 1.8% of their sample population [3]. Bilateral testicular loss commonly follows delay in providing definitive surgical intervention in form of surgery to untwist the spermatic cord followed by fixation of both testis with non absorbable suture material [1, 4]. Mawingiro described testicular loss as being “directly related to delay in surgery and the referral patterns” of health workers [5]. In this paper we explore one surgeon's experiences with a series of cases of testicular torsion to demonstrate the importance of the patient's age in the diagnosis of testicular torsion.

## Methods

This was a surgical audit on a series of cases covering a span of 30 years in Uganda, Kenya, Rwanda, South Africa, Nigeria, and France. The cases included in the study were those in whom the diagnosis was either testicular torsion or orchitis. For each case the following details were captured; age of the individual, country, diagnosis at admission, medical treatment given, findings on surgery, confirmation of diagnosis after surgery and outcome for the patient testis involved.

The information from the patients’ records was kept as a record of surgeries done by the first author and is now used as a case series for secondary analysis in this paper. The information was analyzed using descriptive statistics and non parametric tests whose level of significance was set at 0.05 unless otherwise specified.

## Results

There were 305 patient records seen, with an age range of 9–56 years. There were 195/305 (64%) patients presenting with orchitis while the rest 110/305 (36%) presented with testicular torsion. In 68/305 (23.3%) cases both testicles were involved, while in 111/305 (36.4%), had involvement of the left testis with the rest 126/305 (41.3%) having the right testis affected. There were 62/305 (20.3%) cases that required bilateral fixation, while 195/305 (63.9%) had no fixation done at surgery, the remaining 48/305 (15.7%) ended up with removal of the testis. In 294/303 (97%) cases there was no miss diagnosis compared with 9/303 (3%) with a miss diagnosis. There was an additional 2/305 records for which there were no record of miss diagnosis.

In Table 1 note that there were significant differences in the ages of the patients from the different countries (H (6) = 84.364, p) Figure 1; which shows that testicular torsion is more common under the age of 18 years while orchitis was more common after 18 years of age (Spearmans rho= −0.834, p value > 0.001 one tailed). Further note In Table 1 there are significant differences in diagnosis between the countries (H (6) = 121.8, p <0.001). These differences were significant as shown by a higher incidence of torsion (100%) in France, reducing to 32% in Uganda-2 (J = 15478, z = − 4.488, r = − 0.26). From the same table note that there was a significant increase in the diagnosis of orchitis over time (J= 20201, z = 2.041, r = 0.16).

**Figure 1:** Box plot showing initial diagnosis and age for the different countries where cases presented

**Table 1:** Showing Age and diagnosis made in the different countries

Country	years	N	Age					Diagnosis (number)	
			Mean Age	Std. Deviation	Std. Error	Minimum	Maximum	Ochitis	Torsion
France	1987–1994	48	12.96	2.133	.308	9	17	0	48
Kenya	1981–1982	24	26.42	7.471	1.525	13	40	20	4
Nigeria	1983–1986	52	30.42	8.472	1.175	13	53	51	1
R.S.A	1997–2003	83	27.23	12.668	1.390	9	56	53	30
Rwanda	1995–1996	10	29.40	8.784	2.778	20	52	10	0
Uganda	2003–2011	15	24.87	8.158	2.106	13	40	11	4
Uganda-2	1980–1981	73	23.88	8.071	.945	12	37	50	23
**Total**		**305**	**24.62**	**10.548**	**.604**	**9**	**56**	**195**	**110**

## Discussion

Testicular torsion is a medical emergency requiring quick and urgent action. This is due to the fact that torsion leads to testicular death by ischemia within 6 hours [1]. Beyond the six hours, the chances of saving the testis reduce over the next 48 hours [6]. Given the painful nature of the condition the patient's response is usually rapid with delays being observed at the first contact with the health care system [1, 5, 7]. In this set of case series no note was made of the delays in getting to the health units for definitive management. Other African authors have noted that delays arose when patients received the wrong diagnosis resulting in the management of torsion as orchitis [7, 8]. One of the long term effects of a missed testicular torsion diagnosis for the patient is sterility [9, 10]. This makes having the correct diagnostic knowledge for testicular torsion by the first care giver a very important factor in determining the outcomes of testicular torsion.

Most African authors agree that patients presenting with testicular swelling and below the age of 20–18 years should be managed as testicular torsion while those above this age range as orchitis [1, 4–8]. In this study as summarized in both Table 1 and Figure 1 there is a clear distinction in the age of presentation for orchitis as compared to torsion. This further confirms that age can be used as a rule of thumb in the diagnosis of this condition. The difference between this study and the others is that here the cases were identified from various settings with the same observation. Based on this observation we strongly support the idea proposed by Dwivedi, Joharapurkar and Golhar for an educational intervention to identify patients with torsion using age based algorithms in low resource settings [11].

This was a study on 305 records over a 30 year span of experience by one individual. While it is not possible to rule out bias due to increasing experience, difference in resources and disease patterns from country to country as shown in Table 1, the findings of this study do not seem to affect the age related incidence or the two conditions. A clear example is seen in comparing the observations made in France with those made elsewhere (Figure 1). This is further confirmed by the small effect of time (r = 0.16) for a more frequent diagnosis of orchitis over the years. Thus age remains a valid candidate for differential diagnosis of the two conditions in any setting.

## Conclusion

This paper highlights the importance of age as a diagnostic criterion for the rapid management of testicular torsion. Based on this study we recommend the development of educational interventions that promote the use of age cut offs as a simple diagnostic rule of the thumb in the management of testicular torsion or ochitis by low cadre health workers in the community for low resource settings.
